# Features of a giant cell tumour of the parotid gland: A case report

**DOI:** 10.3892/ol.2013.1462

**Published:** 2013-07-15

**Authors:** CHENG-JUNG WU, PI-HSIUNG WU, SAU-TUNG CHU, WEI-WEN YU, PO-CHUN CHEN

**Affiliations:** 1 Department of Otolaryngology - Head and Neck Surgery, Kaohsiung Veterans General Hospital, Kaohsiung 81362, Taiwan, R.O.C.; 2 Institute of Clinical Medicine, Kaohsiung Medical University, Kaohsiung 80708, Taiwan, R.O.C.; 3 Department of Pathology, Kaohsiung Veterans General Hospital, Kaohsiung 81362, Taiwan, R.O.C.; 4 Department of Dermatology, Kaohsiung Veterans General Hospital, Kaohsiung 81362, Taiwan, R.O.C.; 5 Department of Radiation Oncology, Kaohsiung Veterans General Hospital, Kaohsiung 81362, Taiwan, R.O.C.

**Keywords:** giant cell tumour, parotid gland tumours

## Abstract

A giant cell tumour (GCT) is a benign tumour that commonly arises in the distal end of the long bones. Extraosseous GCTs have been reported in a number of organs, but it is rare for a GCT to present in the parotid gland. Therefore, primary GCTs of the parotid gland (GCTPs) are extremely rare. Although GCTPs have been identified as benign soft-tissue tumours, they have a highly malignant potential and poor prognosis. In the present case, we report a 58-year-old male patient presenting with non-tender mass over the left preauricular area for 11 months. The final pathology report revealed a rare case of a GCTP that was treated by parotidectomy and adjuvant radiation therapy. The patient had no recurrence after 2 years of follow-up.

## Introduction

A giant cell tumour (GCT) is generally considered as a benign tumour originating from the bone. Extraosseous giant cell tumours have been reported in a number of organs, including the temporomandibular joint (1), larynx (2), maxillary sinus (3) and other soft tissues. Primary giant cell tumours of the parotid gland (GCTPs) were first described by Eusebi *et al* in 1984 (4). A GCTP is considered to be extremely rare, with only a few well-documented, histopathologically-confirmed cases previously published in the English literature. In addition, the majority of previous studies have been performed by pathologists and have focused on discussing the histopathological observations of GCTP. The present case report is the first to analyse the treatment policy and prognosis of GCTP. Therefore, the current study presents a rare case of GCTP and a review of the literature in order to improve our understanding of this disease. Written informed consent was obtained from the patient.

## Case report

A 58-year-old male was admitted to Kaohsiung Veterans General Hospital (Kaohsiung, Taiwan) with an 11-month history of a non-tender mass over the left preauricular area with no relevant medical history. A physical examination revealed a painless, hard, elastic mass (4×3 cm) over the left preauricular area. The results of a head and neck examination were within normal limits and facial nerve function was intact. A fine-needle aspiration was performed over the left parotid gland using a 22-gauge needle and the histopathological study was not able to exclude the presence of a malignancy. Subsequent observations by computed tomography showed that a mass (4×3×1.5 cm^3^) was occupying the deep lobe of the left parotid gland (Fig. 1).

The patient received a total parotidectomy due to suspected malignancy. Following confirmation of all the facial nerve branches, the superficial lobe of the left parotid gland was resected and the tumour was exposed (Fig. 2). The tumour (4×3×1.5 cm^3^) was observed to be occupying the deep lobe of the left parotid gland. Following removal of the tumour, the facial nerve trunk and its branches were preserved over the deep lobe of the left parotid gland.

The tumour was sent for histopathological examination by immunohistochemistry. The sections of the specimen were identified as that of a giant cell tumour, composed of uniformly distributed osteoclast-like giant cells, admixed with mononuclear cells and numerous brown hemosiderin-laden macrophages (Fig. 3A). The immunohistochemistry results identified that the osteoclast-like giant and mononuclear cells were positive for CD68 (Fig. 3B) and negative for cytokeratin, S100 and HMB-45.

Following surgery, the patient was referred to the Department of Radiation Oncology (Kaohsiung Veterans General Hospital, Kaohsiung, Taiwan) for adjuvant radiation therapy since surgical margins were not achieved. Treatment consisted of surgical excision associated with adjuvant radiation therapy. No facial palsy was observed following surgery and radiation therapy (6400 cGy, 32 fractions over the tumor bed in the left parotid fossa), and the individual exhibited no recurrence of a neoplasm after 2 years of follow-up.

## Discussion

GCTs are generally considered as benign tumours that originate from the bone. Extraosseous giant cell tumours have been reported in a number of organs, including the temporomandibular joint (1), larynx (2), maxillary sinus (3) and other soft tissues. Primary GCTPs were first described by Eusebi *et al* in 1984 (4), however, due to their rarity, there is an absence of literature that has analysed GCTP and all published material has been case reports. A summary of fifteen case reports, located using PubMed in a search of data up to May 2012, are presented in Table I(4–13). The most common clinical presentation of a GCTP was a non-tender, growing mass over the preauricular area followed by swelling of the parotid gland. The average age at presentation was 62.6 years and ranged between 30 and 92 years. In addition, 19% of patients (3/16) were <50 years old at diagnosis, whereas 56% of patients (9/16) were >60 years old. The male to female ratio was 7:1, indicating a male predilection for GCTPs, an observation that, to the best of our knowledge, has not been previously reported. By contrast, GCTs of the bone had a female predilection.

A GCTP is a rare primary soft-tissue tumour that is pathologically and clinically similar to a GCT of the bone. However, it is recognised as a distinct entity in the World Health Organization Classification of Tumours for soft tissue and bone (14). Although the two tumours may be indistinguishable morphologically, various clinical results and histological features aid in the differentiation between the two. GCTP is biologically more aggressive and, morphologically, may show decreased mitotic activity, a lack of reactive bone formation at the periphery of the tumour and is commonly admixed with a mononuclear component (12). The resected specimen of the patient was identified as a GCT, composed of uniformly distributed osteoclast-like giant cells, admixed with mononuclear cells and exhibiting a lack of bone formation at the periphery of the tumour. The giant cells were large, multinucleated (10–50 nuclei) and shown to be positive for CD68 and negative for cytokeratin, S100 and HMB-45. Mitotic activity measured up to 2/10 HPF, with an absence of atypical mitosis and cytological atypism. The identification of a GCTP should warrant an investigation for a carcinomatous component since this component is likely to be focal and small (12).

Among the 16 patients with available treatment records, the majority received a parotidectomy alone. One patient was managed by a parotidectomy with neck dissection due to cervical lymph node metastasis, and an additional patient received parotidectomy with en bloc resection of the parapharyngeal space tumour due to parapharyngeal invasion. Eight patients were diagnosed with an associated carcinomatous component and were managed by surgery alone. Of these patients, two succumbed to the disease within <28 months. All eight patients who were diagnosed without an associated carcinomatous component remained free of disease and survived. These observations indicate that GCTP patients diagnosed with an associated carcinomatous component exhibit increased mortality rates of up to 25% (2/8).

For the treatment of malignant parotid tumours, parotidectomies and post-operative adjuvant radiation therapy have been used (15). A previous study reported that 59.4% of patients who had received radiation therapy demonstrated a survival benefit (16). A GCTP is considered as a benign soft-tissue tumour, but one with malignant potential. The observations of the current case report indicate that the incidence of an associated carcinomatous component in GCTP is extremely high [50% of patients (8/160)] and is not likely to be due to incidental coexistence (Table I).

The basic treatment for a GCT is extensive resection of the tumour, allowing for a sufficient margin of the surrounding normal tissue (8). A GCT is a radiosensitive tumour and, therefore, radiotherapy is highly effective. Radiotherapy is a reasonable option under conditions where negative surgical margins may only be achieved with increased morbidity or if surgery has been contraindicated (15). The patient presented in the current case report received a total parotidectomy followed by adjuvant radiation therapy due to negative surgical margins. Surgery alone may not be suitable for patients diagnosed with an associated carcinomatous component. A review of the related literature revealed that 25% (2/8) of GCTP patients with a carcinomatous component developed pulmonary metastasis and succumbed to the GCTP (Table I). Among these eight patients, seven did not receive radiation therapy, and the radiation therapy of the single patient who did receive treatment was terminated due to poor tolerance. By contrast, a GCT of the temporomandibular joint may be well managed by complete removal of the tumour alone rather than by complete surgery with combined radiation therapy (1). The results of the present report indicated that a combination of complete surgery and post-operative radiation therapy is the treatment of choice for achieving greater locoregional control and improved cure rates for the treatment of patients with a carcinomatous component or negative surgical margins.

In summary, GCTPs are uncommon benign tumours with a malignant potential. The identification of a GCTP should warrant a diligent search for a carcinomatous component. Complete surgical removal of the tumour is the treatment of choice for a resectable GCTP. In addition, surgery alone has been justified for the management of a GCTP without a carcinomatous component. However, combined radiation therapy is recommended if surgery has been contraindicated, if surgical margins have not been achieved or if GCTP has been diagnosed with an associated carcinomatous component.

## Figures and Tables

**Figure 1:** Computed tomography scan (axial view) of a mass, indicated by the arrow, identified in the parotid gland.

**Figure 2:** Following the complete resection of the superficial lobe of the left parotid gland, the primary tumour, indicated by the arrow, was identified. The tumour occupied the deep lobe of the left parotid gland.

**Figure 3:** (A) Histological and immunophenotypical features of the biopsy specimen. Hematoxylin and eosin staining revealed uniformly distributed osteoclast-like giant cells, indicated by the black arrow, admixed with mononuclear cells, indicated by the white arrow (magnification, ×400). (B) Positive expression of CD68 (magnification, ×200).

**Table I:** Summary of GCTPs from previous studies.

First author (ref.)	Age, years	Gender	Size, cm	Carcinomatous component	Surgery	Radiation therapy	Meta	Follow-up (months)
Eusebi *et al*(4)	30	M	2.2	No	Parotidectomy	No	No	NED (48)
Eusebi *et al*(4)	52	M	1×0.8×0.8	No	Parotidectomy	No	No	NED (48)
Eusebi *et al*(4)	43	M	2×1.5	Ex pleomorphic adenoma	Parotidectomy	No	No	NED (60)
Balogh *et al*(5)	67	M	6×5×4	Infiltrating intraductal	Parotidectomy ductal Ca	RT was stopped due to poor tolerance	P	DWD (28)
Batsakis *et al*(6)	59	M	3×2.5×2.5	High-grade ductal	Parotidectomy	No	No	NED (12)
Batsakis *et al*(6)	92	M	2×1.5×1.5	No	Parotidectomy with en bloc resection of parapharyngeal space tumour	No	No	NED (9)
Ellis *et al*(7)	70	F	NA	No	NA	NA	No	NA
Ellis *et al*(7)	65	M	NA	No	NA	NA	No	NA
Ellis *et al*(7)	73	M	NA	No	NA	NA	No	NA
Itol *et al*(8)	53	M	8×6	No	Parotidectomy	No	No	NA
Grenko *et al*(9)	66	F	5	Carcinomsarcoma with a salivary duct	Parotidectomy	No	P	DWD (13)
Donath *et al*(10)	82	M	1.5	Ex pleomorphic adenoma	NA	No	No	NA
Tse *et al*(11)	75	M	1.1	Salivary duct	Parotidectomy	No	No	NA
Kadivar (12)	75	M	6.5	Salivary duct	Parotidectomy and neck dissection	No	C	NA
Fang *et al*(13)	43	M	7×7×6.5	Salivary duct	Parotidectomy	No	No	NED (12)
Present case	58	M	4×3×1.5	No	Parotidectomy	Yes	No	NED (24)

GCT, giant cell tumour of the parotid gland; RT, radiation therapy; NED, no evidence of disease; Ca, carcinoma; DWD, succumbed to disease; NA, not available; M, male; F, female; meta, metastasis; P, pulmonary metastasis; C, cervical neck lymph node metastasis.

## References

[1] De Benedittis M, Turco M, Petruzzin M, Cortelazzi R (2013). Extra-articular diffuse-type giant cell tumour of the temporomandibular joint. Int J Oral Maxillofac Surg.

[2] Nishimura K, Satoh T, Maesawa C (2007). Giant cell tumor of the larynx: a case report and review of the literature. Am J Otolaryngol.

[3] Hoffman CD, Huntley TA, Wiesenfeld D, Kleid S, Kung IT (1994). Maxillar giant cell tumour associated with Paget’s disease of bone. Int J Oral Maxillofac Surg.

[4] Eusebi V, Martin SA, Govoni E, Rosai J (1984). Giant cell tumor of major salivary glands: report of three cases, one occurring in association with a malignant mixed tumor. Am J Clin Pathol.

[5] Balogh K, Wolbarsht RL, Federman M, O’Hara CJ (1985). Carcinoma of the parotid gland with osteoclastlike giant cells. Immunohistochemical and ultrastructural observations. Arch Pathol Lab Med.

[6] Batsakis JG, Ordonez NG, Sevidal PA, Baker JR (1988). Osteoclast-type giant cell neoplasms of the parotid gland. J Laryngol Otol.

[7] Ellis GL, Auclair PL, Gnepp DR (1991). Surgical pathology of the salivary glands. Major Problems in Pathology Series.

[8] Itoh Y, Taniguti Y, Arai K (1992). A case of giant cell tumor of the parotid gland. Ann Plast Surg.

[9] Grenko RT, Tytor M, Boeryd B (1993). Giant-cell tumor of the salivary gland with associated carcinosarcoma. Histopathol.

[10] Donath K, Seifert G, Röser K (1997). The spectrum of giant cells in tumours of the salivary glands: an analysis of 11 cases. J Oral Pathol Med.

[11] Tse LL, Finkelstein SD, Siegler RW, Barnes L (2004). Osteoclast-type giant cell neoplasm of salivary gland. A microdissection-based comparative genotyping assay and literature review: extraskeletal ‘giant cell tumor of bone’ or osteoclast-type giant cell ‘carcinoma’?. Am J Surg Pathol.

[12] Kadivar M, Nilipour Y, Sadeghipour A (2007). Osteoclast-like giant-cell tumor of the parotid with salivary duct carcinoma: case report and cytologic, histologic, and immunohistochemical findings. Ear Nose Throat J.

[13] Fang X, Hicks DG, Hicks W, Zhang S (2009). Osteoclastlike giant cell tumor of the salivary gland. Ann Diagn Pathol.

[14] Barnes L, Eveson JW, Reichart P, Sidransky D (2005). World Health Classification of Tumours. Pathology and Genetics of Head and Neck Tumours.

[15] Lin CC, Tai MH, Huang CC (2008). Parotid tumors: a 10-year experience. Am J Otolaryngol.

[16] Bhattacharyya N, Fried MP (2005). Determinants of survival in parotid gland carcinoma: a population-based study. Am J Otolaryngol.

